The article "Expression of lncRNA MALAT1 through miR-144-3p in Osteoporotic Tibial Fracture Rats and Its Effect on Osteogenic Differentiation of BMSC under Traction" was retracted in 2023. Reasons: signs of a paper mill; suspected computer-generated content; unreliable results or conclusions; concerns about the data.

# Expression of lncRNA MALAT1 through miR-144-3p in Osteoporotic Tibial Fracture Rats and Its Effect on Osteogenic Differentiation of BMSC under Traction

**DOI:** 10.1155/2022/2590055

**Published:** 2022-07-05

**Authors:** Shiyong Ling, Tao Xu, Jingchuan Sun, Chen Yan, Bo Lv, Hua Wang, Hong Zhao, Kai Huang

**Affiliations:** ^1^Department of Orthopedic Surgery, Zhabei Central Hospital, Jing'an, Shanghai 200070, China; ^2^Department of Orthopedic Surgery, No. 906 Hospital of the People's Liberation Army, Ningbo, Zhejiang 315040, China; ^3^Department of Orthopedic Surgery, Spine Center, Changzheng Hospital, Second Military Medical University, Shanghai 200003, China

## Abstract

**Objective:**

To investigate the expression of lncRNA MALAT1 and miR-144-3p in osteoporotic (OP) tibial fracture rats and analyze their targeting relationship and effects on the osteogenic differentiation of bone marrow mesenchymal stem cells (BMSC) under traction.

**Methods:**

The OP tibial fracture model was established, and the rats were divided into a sham group and a model group. The tibial tissue of these rats was taken. BMSC of cultured rats with good growth was purchased and grouped according to the presence or absence of transfection of si-MALAT1 and miR-144-3p-mimic. The expression of MALAT1 and miR-144-3p in each group was detected. The bioinformatics website and double luciferase were used to predict the targeting relationship between MALAT1 and miR-144-3p and to detect the expression of genes related to bone differentiation (collagen I, osteocalcin (OCN), osteopontin (OPN), and alkaline phosphatase (ALP)) of each component, and ALP staining and AR staining were used to detect the formation of BMSC calcium nodules.

**Results:**

The levels of ALP and TRAP in the model group were higher than that in the sham group (*P* < 0.05). qRT-PCR results showed that the relative expression level of MALAT1 in the model group was higher than that in the sham group, and the relative expression level of miR-144-3p was lower than that in the sham group (*P* < 0.05). MALAT1 has a targeting relationship with miR-144-3p. qRT-PCR results showed that the relative expression level of MALAT1 in the tension-MSC group was higher than the MSC group, and the relative expression level of miR-144-3p was lower than the MSC group (*P* < 0.05). The expressions of collagen I, OCN, OPN, and ALP proteins in the si-MALAT1 group were higher than those of the si-NC group (*P* < 0.05). The results of ALP staining showed that BMSCs of the si-MALAT1 group had stronger osteogenic differentiation capacity and higher ALP activity than those of the si-NC group. The results of AR staining showed that compared with the si-NC group, the mineralization degree of cells in the si-MALAT1 group was higher, the number of calcium nodules was more, and the cells were more deeply stained. The expressions of collagen I, OCN, OPN, and ALP proteins in the miR-144-3p-mimic group were higher than the mimic-NC group (*P* < 0.05). ALP staining results showed that BMSCs in the miR-144-3p-mimic group had strong osteogenic differentiation capacity and high ALP activity compared with the mimic-NC group. The results of AR staining showed that, compared with the mimic-NC group, the mineralization degree of cells in the miR-144-3p-mimic group was higher, the number of calcium nodules was more and the cells were more deeply stained.

The article "Expression of lncRNA MALAT1 through miR-144-3p in Osteoporotic Tibial Fracture Rats and Its Effect on Osteogenic Differentiation of BMSC under Traction" was retracted in 2023. Reasons: signs of a paper mill; suspected computer-generated content; unreliable results or conclusions; concerns about the data.

**Conclusion:**

In the OP rat model with the tibial fracture, the expression of MALAT1 is upregulated and that of miR-144-3p is downregulated. MALAT1 has a targeting relationship with miR-144-3p, and downregulation of MALAT1 and upregulation of miR-144-3p can promote the osteogenic differentiation of BMSC under traction.

## 1. Introduction

Osteoporosis (OP), one of the common bone metabolic diseases in clinic, is characterized by changes in the bone microstructure and reduction in bone mass per unit volume, which is more common in elderly men and postmenopausal women [1, 2]. OP can easily reduce the strength and increase the brittleness of bones and greatly increase the possibility of fractures in patients. In daily life and work, fractures may occur under the action of a slight external force, which are prone to occur in the forearm, spine, hip, and other areas. As people age, it leads to the loss of a large amount of calcium in the body, the body's bone mineral density will be reduced, and the risk of the fracture is becoming more and more big [3, 4]. Once secondary fractures occur in the elderly, they need to stay in bed and rest, and then, there will appear various complications, including pulmonary infection and bedsore. Because of the insufficient local blood supply, fractures are difficult to heal, which may cause disability and threaten the life and health of the elderly. As the most serious consequence of OP, tibial fracture will bring severe living burden and economic burden to patients [5, 6]. Bone marrow mesenchymal stem cells (BMSC) are stromal cells with the potential of continuous self-renewal and multidirectional differentiation. Under specific induction conditions, these cells can differentiate into osteoblasts, chondrocytes, and adipocytes [7, 8]. The differentiation regulation of BMSCs is involved in the regulation of a variety of molecular pathways, showing a good potential in the stem cell therapy of osteogenic diseases [9, 10]. lncRNA not only plays an important role in a variety of tumor tissues but also plays a regulatory role in bone growth and differentiation. MALAT1 is one of the important members of the lncRNA family. The original study mainly focused on its relationship with tumors [11, 12]. Other studies have shown that MALAT1 can promote the survival and angiogenesis of BMSC [13, 14]. miR-144-3p is involved in the proliferation and differentiation of a variety of cancer cells, and it is a recognized anticancer factor [15–17]. Kim et al. [18] detected that the expression of miR-144-3p was decreased in osteogenic differentiation, indicating that miR-144-3p might be involved in the differentiation of mesenchymal stem cells. The purpose of this study was to investigate the expression of lncRNA MALAT1 and miR-144-3p in OP tibial fracture rats and analyze the targeting relationship between the two and their effects on the osteogenic differentiation of BMSC under traction.

The article "Expression of lncRNA MALAT1 through miR-144-3p in Osteoporotic Tibial Fracture Rats and Its Effect on Osteogenic Differentiation of BMSC under Traction" was retracted in 2023. Reasons: signs of a paper mill; suspected computer-generated content; unreliable results or conclusions; concerns about the data.

## 2. Materials and Methods

### 2.1. Animals

8 SPF-grade female SD rats were selected, all purchased from Kai Student Biology Technology (Shanghai) Co., Ltd. Feeding environment: temperature, 22° ± 2°C; illumination, 150–200 lx; 12 h/12 h alternation of light and shade; relative humidity, 50–60%; and free diet. The rats were divided into a sham group and a model group. Bilateral ovaries of the model group were removed, while the exposed ovary of the sham group was not removed. All animal experiments are conducted in accordance with the National Institutes of Health, “Guidelines for the Care of Laboratory Animals,” and the regulations of our hospital's ethics committee.

### 2.2. Experimental Methods

The OP model was established [19], and bilateral oophorectomy was performed from the back under anesthesia with ketamine hydrochloride (20 mg/kg). The blood levels of ALP and TRAP in rats were detected by ELISA, and kits were purchased from Shanghai Enzymolysis Biotechnology Co., Ltd. The tibial fracture model was established after passing the test. Establishment of the tibial fracture model [20]: the left posterior limb of the rat was properly fixed on the anvil groove of the compression experiment of the universal mechanical experimental machine. After the computer showed that the compressive force reached the peak, the blunt impact knife perpendicular to the long diameter of the tibia of the rat at the speed of 10 cm/s struck the tibia of the rat. Depilation and disinfection of the rat fracture site: a 1.0 mm Kirschner wire was vertically inserted into both sides of the broken end of the fracture to correct the force line of the lower limb, and the external fixator was fixed firmly. X-ray fluoroscopy showed that the fracture was aligned, and the external fixation was in place, confirming the success of modeling. Tibial tissues were taken, and the expressions of MALAT1 and miR-144-3p were detected by qRT-PCR.

The article "Expression of lncRNA MALAT1 through miR-144-3p in Osteoporotic Tibial Fracture Rats and Its Effect on Osteogenic Differentiation of BMSC under Traction" was retracted in 2023. Reasons: signs of a paper mill; suspected computer-generated content; unreliable results or conclusions; concerns about the data.

BMSC of cultured rats with good growth were purchased, digested with 0.25% trypsin solution, and then inoculated with *l* × 10^5^ cm^−2^ solution on a 6-well elastic silica gel afterburner. After standing for culture for 48 h, 80%–90% of the samples were fused. Subsequently, using the Flexercell in vitro cell mechanics loading device, BMSC were harvested and induced into osteoblastic differentiation in vitro under the traction force with a frequency of 1 Hz and a deformation rate of 18% for 30 min, twice a day for 5 days. Subgroups: the control group (untransfected BMSC), the si-NC group (transfected with MALAT1 inhibitor negative control), the si-MALAT1 group (transfected with MALAT1 inhibitor), the mimic-NC group (transfected with miR-144-3p mimic negative control), and the miR-144-3p-mimic group (transfected with miR-144-3p mimic). The cell differentiation was detected after BMSC was transfected with si-MALAT1 and miR-144-3p mimics. The expressions of osteogenic differentiation related genes (collagen I, osteocalcin (OCN), osteopontin (OPN), and alkaline phosphatase (ALP)) were detected. The formation of calcium nodules and lipid droplets in BMSC was detected by ALP staining and ARS staining.

qRT-PCR analysis: total RNA was extracted by the trizol method and reversely transcribed into complementary DNA. qRT-PCR detection was performed on the computer according to the reagent instructions. Primer sequences: MALAT1 upstream: 5′-CAGACCACCACAGGTTTACAG-3′ and downstream: 5′-AGACCATCCCAAAATGCTTCA-3′; miR-144-3p upstream: 5′-CTCTATCCAAAACAGGCCGC-3′ and downstream: 5′-TTTACATCCCCAAGGCCCAT-3′. The internal reference was GAPDH, and every three wells were taken as a sample to obtain the Ct value of each group.

#### 2.2.1. Western Blot Analysis

The protein was quantified by the extraction of the total protein BCA method. Sodium dodecyl sulfate polyacrylamide gel electrophoresis (SDS-PAGE) gel electrophoresis was performed. The membrane was transformed for 1 h in ice bath, sealed at room temperature by BSA and incubated overnight at 4°C with primary antibody. The membrane was washed for 3 times, 10 min each. The second antibody was incubated at room temperature, and the membrane was washed for 3 times, 10 min each. An electrochemical luminescent substrate developing solution was added, and finally, a picture was taken on a gel imaging instrument.

The formation of calcium nodules in BMSC was detected by ALP staining and alizarin red (AR) staining. ALP staining: the BCIP/NBT alkaline phosphatase chromogenic kit purchased from Shanghai Biyuntian Biotechnology Co., Ltd., was used for detection, and the kit instructions were followed. Few drops of No.1 solution was added dropwise to the cell climbing sections, and the sections were fixed at room temperature for 1 min, rinsed for 2 min, and dried. After few drops of action solution were added, the samples were incubated in a wet box at 37°C for 2 h and rinsed for 2 min. Then, few drops of No.5 solution was added dropwise, counterstained for 5 min, rinsed for 2 min, dried, and photographed with a microscope. AR staining: the cells were transferred to the slide, fixed in 95% ethanol for 10 min, and rinsed with double distilled water for three times and then incubated in 0.1% alizarin red staining solution (purchased from Beijing Solebo Technology Co., Ltd.) for 30 min. The sections were washed with distilled water, dried, sealed, and photographed under a microscope.

The article "Expression of lncRNA MALAT1 through miR-144-3p in Osteoporotic Tibial Fracture Rats and Its Effect on Osteogenic Differentiation of BMSC under Traction" was retracted in 2023. Reasons: signs of a paper mill; suspected computer-generated content; unreliable results or conclusions; concerns about the data.

A dual-luciferase reporter assay: the binding sites of miR-144-3p and MALAT1 were analyzed using Jefferson prediction website, and the targeting relationship between MALAT1 and miR-144-3p was verified by a dual-luciferase reporter assay. According to the binding sequence of the 3′UTR region of MALAT1 to miR-144-3p, the synthetic target sequence and the mutant sequence were designed, respectively. Relative luciferase activity = firefly luciferase activity/renin luciferase activity.

### 2.3. Statistical Methods

With SPSS22.0 statistical software, the data was expressed as (mean ± SD), and variance analysis and the LSD-t test showed that the difference was statistically significant with *P* < 0.05.

## 3. Results

### 3.1. OP Establishment of the Tibial Fracture Model in Rats

Serum ALP and TRAP levels in the experimental group were higher than that in the sham group (*P* < 0.05) as shown in Figure 1.

### 3.2. Expression of MALAT1 and miR-144-3p in Tibial Tissue of OP Model Rats

qRT-PCR results showed that the relative expression level of MALAT1 in the experimental group was higher than that in the sham group, and the relative expression level of miR-144-3p was lower than that in the sham group (*P* < 0.05), as shown in Figure 2.

### 3.3. Relationship between MALAT1 and miR-144-3p

The bioinformatics website predicted that MALAT1 was a direct target of miR-144-3p, and the results of the dual-luciferase reporter gene test showed that transfection of miR-144-3p-mimic reduced the luciferase activity of the wild-type MALAT1 3′UTR construct (*P* < 0.05), as shown in Figure 3.

### 3.4. Expression of MALAT1 and miR-144-3p in Osteogenic Differentiation

qRT-PCR results showed that the relative expression level of MALAT1 in the tension-MSC group was higher than the MSC group, and the relative expression level of miR-144-3p was lower than the MSC group (*P* < 0.05), as shown in Figure 4.

The article "Expression of lncRNA MALAT1 through miR-144-3p in Osteoporotic Tibial Fracture Rats and Its Effect on Osteogenic Differentiation of BMSC under Traction" was retracted in 2023. Reasons: signs of a paper mill; suspected computer-generated content; unreliable results or conclusions; concerns about the data.

### 3.5. Inhibiting the Effect of MALAT1 on the Osteogenic Differentiation of BMSC under Traction

The expressions of collagen I, OCN, OPN, and ALP proteins in the si-MALAT1 group were higher than those of the si-NC group (*P* < 0.05). The results of ALP staining showed that BMSCs of the si-MALAT1 group had stronger osteogenic differentiation capacity and higher ALP activity than those of the si-NC group. The results of AR staining showed that, compared with the si-NC group, the mineralization degree of cells in the si-MALAT1 group was higher, the number of calcium nodules was more, and the cells were more deeply stained, as shown in Figure 5.

### 3.6. Effect of Upregulation of miR-144-3p on Osteogenic Differentiation of BMSC under Traction

The expressions of collagen I, OCN, OPN, and ALP proteins in the miR-144-3p-mimic group were higher than the mimic-NC group (*P* < 0.05). ALP staining results showed that BMSCs in the miR-144-3p-mimic group had strong osteogenic differentiation capacity and high ALP activity compared with the mimic-NC group. The results of AR staining showed that, compared with the mimic-NC group, the mineralization degree of cells in the miR-144-3p-mimic group was higher, the number of calcium nodules was more, and the cells were more deeply stained, as shown in Figure 6.

## 4. Discussion

Osteoporosis is a chronic disease caused by the dynamic balance and imbalance of bone metabolism in bones, resulting in the decline of bone mass and destruction of bone microstructures in unit structures. The weakened bone biomechanics of patients is likely to cause fractures, which has caused great pain to patients. When the activity of osteoclasts is greater than that of osteoblasts, it will lead to bone degenerative diseases, such as osteoporosis [21, 22]. BMSC have multi-directional differentiation potential. Promoting their differentiation into osteoblasts can promote bone formation and correct bone metabolism imbalance, playing an important role in the treatment of bone degenerative diseases [23, 24]. miRNAs can recognize multiple osteogenesis-related mRNAs through incomplete complementary pairing and directly regulate the expression of this type of mRNAs to participate in the body's osteogenic differentiation process. It has been reported that the expression of miR-125b is significantly decreased in the differentiation of mouse ST2 osteoblasts, and downregulation of miR-125b can promote the BMP4-induced differentiation of T2 osteoblasts [25]. In BMSCs, miR-218 interacts with a Wnt pathway and positively regulates the process of osteogenic differentiation in BMSCs [26].

The article "Expression of lncRNA MALAT1 through miR-144-3p in Osteoporotic Tibial Fracture Rats and Its Effect on Osteogenic Differentiation of BMSC under Traction" was retracted in 2023. Reasons: signs of a paper mill; suspected computer-generated content; unreliable results or conclusions; concerns about the data.

MALAT1 is a kind of lncRNA, which has no protein coding function, but can mediate transcription regulation and protein posttranslation modification. The lack of expression will result in the loss of protein coding ability, and it can regulate multiple genes to affect bone metabolism, for example, it upregulates the expression of osterix protein to promote osteoblast proliferation and differentiation and downregulates RANKL to inhibit osteoclast activation [27, 28]. MALAT1, an lncRNA first found in lung adenocarcinoma, can mediate the occurrence and development of a variety of bone tumors [29, 30]. In this study, qRT-PCR results showed that the relative expression level of MALAT1 in the model group was higher than that in the sham group, and the relative expression level of MALAT1 in the traction MSC group was higher than that in the MSC group. These results indicated that the expression of MALAT1 was upregulated in the OP rat model of the tibial fracture. The results of this study also showed that compared with the si-NC group, the expressions of collagen I, OCN, OPN, and ALP proteins in the si-MALAT1 group were higher, and the osteogenic differentiation ability of BMSCs was stronger, ALP activity was higher, the degree of cell mineralization was higher, the number of calcium nodules was more, and the cells were deeply stained. These results indicated that lncRNA MALAT1 could regulate the osteogenic differentiation of BMSC.

In order to study the relationship between lncRNA MALAT1 and miR-144-3p, the bioinformatics website has predicted that MALAT1 is the direct target of miR-144-3p. The results of dual-luciferase reporter gene detection showed that transfection of miR-144-3p-mimic reduced the luciferase activity of the wild-type MALAT1 3′UTR construct. All these have fully illustrated the targeting relationship between MALAT1 and miR-144-3p. miR-144-3p is derived from the miR-144/451 cluster on chromosome 11 and can play a role in a variety of tumor or cancer cells. Their inhibitory effect on cell proliferation has also been found in osteosarcoma cells, and by inhibiting cell proliferation, miRNAs are able to inhibit cell osteogenic differentiation because of a dynamic balance between cell proliferation and osteogenic differentiation [31, 32]. In this study, qRT-PCR results showed that the relative expression level of miR-144-3p in the model group was lower than that in the sham group, and the relative expression level of miR-144-3p in the tension-MSC group was lower than the MSC group. These results indicated that the expression of miR-144-3p was downregulated in the OP rat model of the tibial fracture. The results of this study also showed that compared with the mimic-NC group, the miR-144-3p-mimic group had higher protein expressions of collagen I, OCN, OPN, and ALP. BMSCs had stronger osteogenic differentiation ability, higher ALP activity, higher degree of cell mineralization, more calcium nodules, and deeper cell staining. These results indicated that miR-144-3p could regulate the osteogenic differentiation of BMSC.

The article "Expression of lncRNA MALAT1 through miR-144-3p in Osteoporotic Tibial Fracture Rats and Its Effect on Osteogenic Differentiation of BMSC under Traction" was retracted in 2023. Reasons: signs of a paper mill; suspected computer-generated content; unreliable results or conclusions; concerns about the data.

## 5. Conclusion

In the OP tibial fracture rat model, MALAT1 expression was upregulated, and miR-144-3P expression was downregulated. MALAT1 has a targeting relationship with miR-144-3p, and downregulation of MALAT1 and upregulation of miR-144-3p can promote the osteogenic differentiation of BMSC under traction.

## Figures and Tables

**Figure 1:** OP establishment of the tibial fracture model in rats. Note: compared with the sham group, ^*∗*^*P* < 0.05.

**Figure 2:** Expression of MALAT1 and miR-144-3p in tibial tissue of OP model rats. Note: compared with the sham group, ^*∗*^*P* < 0.05.

**Figure 3:** Relationship between MALAT1 and miR-144-3p. Note: compared with the mimic-NC group, ^*∗*^*P* < 0.05.

**Figure 4:** Expression of MALAT1 and miR-144-3p in osteogenic differentiation. Note: compared with the MSC group, ^*∗*^*P* < 0.05.

**Figure 5:** Inhibiting the effect of MALAT1 on the osteogenic differentiation of BMSC under traction.

**Figure 6:** Effect of upregulation of miR-144-3p on osteogenic differentiation of BMSC under traction.

## Data Availability

The data generated and/or analyzed during the current study are available from the corresponding authors upon request.
